The article "Analysis of Current Situation and Influencing Factors of Psychological Distress in Patients with Lung Cancer during Perioperative Period" was retracted in 2023. Reasons: unreliable results or conclusions; concerns about the data; concerns about the peer review; concerns about the citations.

# Analysis of Current Situation and Influencing Factors of Psychological Distress in Patients with Lung Cancer during Perioperative Period

**DOI:** 10.1155/2022/1925668

**Published:** 2022-07-12

**Authors:** Xin He, Na Zhang, Lu Liu, Yan Liu

**Affiliations:** Department of Thoracic Surgery, National Cancer Center, National Clinical Research Center for Cancer, Cancer Hospital, Chinese Academy of Medical Sciences and Peking Union Medical College, Beijing 100021, China

## Abstract

**Objective:**

To explore the degree of psychological distress in patients with lung cancer during the perioperative period and analyze its influencing factors.

**Method:**

A cross-sectional survey was conducted on 372 perioperative patients with lung cancer admitted to our hospital by a convenience sampling method using general data collection and psychological pain thermometer scores.

**Results:**

The psychological distress score of 372 patients with lung cancer in the perioperative period was 4.10 ± 2.88. The psychological distress of patients was related to physical problems, practical problems, medical expenses, and family communication problems. Logistic regression analysis showed that gender, economic burden caused by disease, child care, lack of interest in daily activities, and anxiety were the main factors affecting the degree of suffering of lung cancer patients.

**Conclusion:**

The proportion of perioperative lung cancer patients with a psychological distress score ≥4 points was 55.6%, and more than half of the perioperative patients with lung cancer had a moderate level of psychological distress. Medical staff should pay attention to the management of the psychological distress of patients with lung cancer during the perioperative period, help patients solve practical problems in the process of cancer treatment, strengthen society's attention to female lung cancer patients, and establish a comprehensive cancer public welfare organization group.

## 1. Introduction

According to the latest statistics released by the National Cancer Center of China in March 2022, as of 2020, there will be 9.96 million cancer deaths worldwide, including 1.8 million lung cancer deaths, ranking first in cancer deaths. Far more than other cancer types, up to 710,000, accounting for 23.8% of the total cancer deaths [1]. With increasing morbidity and mortality, lung cancer has clearly become a common cause of global public health threats. At present, perioperative treatment of lung cancer (preoperative neoadjuvant therapy and postoperative adjuvant therapy), as an important adjuvant method for surgery, has become an increasingly important part of the whole management of non-small-cell lung cancer (NSCLC). With the development of perioperative treatment methods to bring better efficacy and survival benefits to patients, there are also related adverse reactions such as delayed surgery, loss of surgical opportunities, and risk of death [2]. Therefore, patients with lung cancer in the perioperative period suffer from a series of psychological pressures when faced with problems such as surgical methods, treatment effects, and postoperative rehabilitation [3]. Along with the shift in biomedical paradigms, in addition to cancer diagnosis and treatment, the patient's own mental health is also considered to be a very important factor affecting prognosis. Psychological distress is a common mental health problem in lung cancer patients. It is a common emotional response of patients to cancer diagnosis and treatment. This response runs through the entire trajectory of the disease and may affect the prognosis of the patient. [4]. The Distress Management Group of The National Comprehensive Cancer Network (NCCN) [5] defines the broad concept of psychological distress as “a multifactorial unpleasant emotional experience of psychosocial and/or psychiatric nature that may interfere with the patient's ability to effectively deal with cancer, its physical symptoms, and treatment.” Numerous studies have found that psychological distress is associated with poor quality of life and disease outcomes and that patients who experience severe distress may be at risk of suicide [6–8]. Russet et al. [9] mentioned that higher psychological distress increases the risk of cancer. Furthermore, these common emotional experiences of vulnerability, sadness, and fear have been extended to disabling problems such as depression, anxiety, panic, social isolation, and mental crisis [10]. A previous cross-sectional study of cancer patients found that at 1 year after surgery, 64% of survivors experienced depression and 80% expressed fear of death and metastasis [11], and these feelings may lead to discontinuation of subsequent chemotherapy or radiation therapy after surgery. Studies have shown that the detection rate of psychological distress in lung cancer patients is the highest. Some data show that the detection rate of psychological distress in Chinese lung cancer patients is 48.3% [12]. Negative effects of high-intensity pain on patients with perioperative lung cancer include reduced adherence to treatment plans, dissatisfaction with overall care, decreased quality of life, and even lower survival rates. Therefore, this study aims to fully understand the current situation of psychological distress in patients with lung cancer in the perioperative period and analyze its influencing factors so as to facilitate clinical treatment and nursing in the future. At the same time, it provides a reference for the screening and evaluation of psychological distress in patients with lung cancer in the perioperative period and the formulation of intervention measures.

The article "Analysis of Current Situation and Influencing Factors of Psychological Distress in Patients with Lung Cancer during Perioperative Period" was retracted in 2023. Reasons: unreliable results or conclusions; concerns about the data; concerns about the peer review; concerns about the citations.

## 2. Materials and Methods

### 2.1. Research Objects

372 perioperative patients with lung cancer who were hospitalized in the Department of Thoracic Surgery, Chinese Academy of Medical Sciences Cancer Hospital from July 2021 to January 2022 during the perioperative period were selected as the research subjects. Inclusion criteria: (1) Age ≥18 years old; (2) confirmed as lung cancer by imaging and histopathology; (3) those who are conscious and able to answer questions correctly; (4) know their condition and diagnosis; (5) informed consent to participate in this researcher voluntarily; and (6) voluntary participation in the informed consent of the researcher. ECOG score of 0 to 1, expected survival ≥3 months. Exclusion criteria: (1) severe mental illness or cognitive impairment; (2) those who gave up or postponed surgical treatment in the middle; (3) those who have received relevant treatment and may affect the effect index observers; and (4) other physiological or pathological conditions accompanied by observation and judgment of influencing effect indicators.

## 3. Methods

### 3.1. Survey Tools

#### 3.1.1. Self-Designed General Information Questionnaire

This includes sociodemographic information such as age, gender, educational level, occupation, and per capita monthly income of the family, and disease-related information such as admission diagnosis, number of cases, and number of lesions.

*(1) Psychological Distress Management Screening Tool*. The distress management screening measure (DMSM) is recommended by the National Comprehensive Cancer Network (NCCN) [13] and consists of two parts: (1) distress thermometer (DT), using 0–10 to indicate the degree of psychological distress, which is marked by the patient according to the average distress level experienced in the past 1 week. 0–3 is mild psychological distress; 4–6 is moderate psychological distress; 7–10 is severe psychological distress; (2) problem list (PL), including various problems encountered by cancer patients after illness, a total of 5 dimensions and 53 questions: physical problems (3) family practical problems (4) emotions questions (5) family questions (6) spiritual/religious questions. The scale is evaluated by closed question and answer. The overall Cronbach's coefficient of the scale was 0.9481.

### 3.2. Survey Methods

This questionnaire is issued during the hospitalization of lung cancer patients. According to the inclusion and exclusion criteria, the star QR code of the questionnaire will be issued to the lung cancer patients who meet the requirements. The patients will scan the code to fill in the questionnaire by themselves and fill it in anonymously. The first page of the questionnaire is explained in a unified guide. Fill out the requirements.

The article "Analysis of Current Situation and Influencing Factors of Psychological Distress in Patients with Lung Cancer during Perioperative Period" was retracted in 2023. Reasons: unreliable results or conclusions; concerns about the data; concerns about the peer review; concerns about the citations.

### 3.3. Ethical Review

This study has been approved by the Ethics Committee of the National Cancer Center/Peking Union Medical College Cancer Hospital, Chinese Academy of Medical Sciences (approval number: 21/018–2689).

### 3.4. Quality Control

Before distributing the questionnaires, the distribution personnel will be trained uniformly through group meetings to make them understand the content of the questionnaires. In the process of distributing the questionnaires, the purpose and significance of this study were explained to the patients, and their informed consent was signed. Questions from the patient's family members were answered in a timely manner during the questionnaire filling process. In order to ensure the authenticity and reliability of the survey results, a time limit for answering questions on WeChat is set, and no missing items can be filled in before submission to ensure the quality of the returned questionnaires.

### 3.5. Statistical Analysis

SPSS20.0 statistical software was used for statistical analysis of the data. The enumeration data, gender, age, smoking, etc., were expressed by frequency (cases), and the measurement data, psychological pain thermometer, and question list scores were expressed as mean ± standard deviation (*x̅* ± *s*) express. *χ*^2^-Test was used to analyze the categorical variables. The bivariate correlation analysis was conducted by the Spearman test, and influencing factors were analyzed by logistic regression analysis. *P* < 0.05 means the difference is statistically significant.

## 4. Results

### 4.1. Overview of Psychological Pain Scores of All Patients

The psychological distress score of lung cancer patients in this study was 4.10 ± 2.88, of which 207 patients had a distress score of ≥4, accounting for 55.6%, as shown in Table 1.

### 4.2. General Information of Perioperative Patients with Lung Cancer

A total of 372 lung cancer patients were collected in this study, including 142 males and 230 females. The results of univariate analysis showed that there were statistically significant differences among patients with different genders, family relationships, economic burden caused by disease, current status, and incidence of disease (*P* < 0.05), as shown in Table 2.

### 4.3. Correlation Analysis of Psychological Distress and Clinical Factors in Perioperative Patients with Lung Cancer

The results of correlation analysis showed that the patient's psychological pain and physical problems (appearance changes, surgical scars, breathing conditions, urination changes, indigestion, memory/attention, nausea/nausea, etc.) were related. Practical problems (caring for children, housekeeping (housekeeping), daily economic situation of the family); problems with medical expenses (inconvenient travel, work/study, disrupted daily life); emotional problems (depression, fear, sadness, etc.); and family communication problems (communication with parents) were related to these factors as shown in Table 3.

The article "Analysis of Current Situation and Influencing Factors of Psychological Distress in Patients with Lung Cancer during Perioperative Period" was retracted in 2023. Reasons: unreliable results or conclusions; concerns about the data; concerns about the peer review; concerns about the citations.

### 4.4. Logistic Regression Analysis of Psychological Distress Scores in Perioperative Patients with Lung Cancer

The variables with statistically significant differences (*P* < 0.05) in the univariate and correlation analysis were subjected to multivariate logistic regression analysis. The results showed that gender, economic burden of disease, child care, lack of interest in daily activities, and anxiety were the main factors affecting psychological distress as shown in Tables 4 and 5.

## 5. Discussion

### 5.1. Status of Psychological Distress in Patients with Lung Cancer during the Perioperative Period

In this study, the psychological distress score of lung cancer patients was 4.10 ± 2.88, of which 207 patients had a distress score of ≥4, accounting for 55.6%, which was higher than the results of Chen Huan [12] (48.3%) and others. It shows that more than half of lung cancer surgery patients in the perioperative period are in moderate psychological distress, which may be related to factors such as patients' cognition of the disease, disease severity, and different treatment stages. It is suggested that clinical nurses should pay more attention to the psychological distress of patients with lung cancer in the perioperative period. Clinical nurses are on the front line of dealing with the psychological distress of patients, and both nurses and patients can fully communicate with each other under the condition of mutual respect, including how to communicate the progress of the disease, adverse reactions, and treatment decisions. At the same time, the patient's difficult situation should be understood, and psychological distress should be informed as a normal and expected response. At the same time, it is also necessary to ensure that patients can obtain relevant social support information, such as support teams, conference calls, and helplines, to help perioperative lung cancer patients reduce psychological pain so that they can actively cooperate with surgical treatment and achieve better postoperative rehabilitation results.

The article "Analysis of Current Situation and Influencing Factors of Psychological Distress in Patients with Lung Cancer during Perioperative Period" was retracted in 2023. Reasons: unreliable results or conclusions; concerns about the data; concerns about the peer review; concerns about the citations.

### 5.2. Univariate Analysis of Psychological Distress in Patients with Lung Cancer during the Perioperative Period

The results of univariate analysis showed that there were statistically significant differences in gender, family relationship, economic burden caused by the disease, current status, and incidence of different lung cancer patients in the perioperative period. Among them, gender and economic burden caused by disease are included in the final regression equation. Therefore, the results of family relationships, current status, and incidence of disease that are not included in the regression equation are discussed here. Patients with good family relationships have lower psychological pain scores. A good family atmosphere can bring comfort to patients, reduce loneliness and fear, and help patients view the disease more positively, optimistically, and correctly, thereby reducing their psychological pain feelings. It is suggested that as family members, we should pay attention to the role of family support. Cancer patients will have many needs limited after the disease, which will affect their emotions and behaviors. Family members should understand the patient's psychological changes as soon as possible, carefully observe the patient's needs, meet the patient's reasonable needs, and provide psychological and behavioral help and guidance [14]. The psychological pain of postoperative patients is higher than that of preoperative patients, which is consistent with the conclusion of previous research [15]. The possible reason is that the patient has undergone surgical treatment, and the persistent symptoms such as pain, fatigue, and other complications after surgery have caused his body to suffer. In a relatively weak period, and faced with problems such as follow-up rehabilitation, radiotherapy and chemotherapy, recurrence, and risk of metastasis [16], their psychology is also in the unstable period of disease development. Therefore, under the influence of both physical and psychological aspects, postoperative psychological distress experiences are more severe, prominent, and complex. Studies have shown that self-management has a positive impact on patients' postoperative recovery, can reduce psychological stress and improve their quality of life [17]. In the future, clinical nurses can further explore ways of self-management of postoperative patients to help them relieve psychological pain. The psychological distress score of patients with initial lung cancer is higher than that of patients with recurrence, which is consistent with the research results of Tang Lili [18] and others. According to the psychological activity staging of cancer patients proposed by American health psychologist Kubler-Ross, the first-episode patients are in the stage of denial; that is, when they first learn that they have cancer, the vast majority of patients simply cannot accept this fact. Due to the high level of psychological distress caused by emergencies, the relapsed patients have experienced previous treatment, have gradually accepted the disease, and their psychological adaptation level has been improved, so the degree of distress is lower than before. This also suggests that medical staff should pay attention to the changes in the psychological level of patients in different stages of the disease, especially the psychological state of patients in the early stages of the disease, help them to better complete the psychological transition, and provide rehabilitation care for the psychological stages of patients.

The article "Analysis of Current Situation and Influencing Factors of Psychological Distress in Patients with Lung Cancer during Perioperative Period" was retracted in 2023. Reasons: unreliable results or conclusions; concerns about the data; concerns about the peer review; concerns about the citations.

### 5.3. Analysis of Related Factors of Psychological Distress in Patients with Lung Cancer during the Perioperative Period

In this study, the factors related to the psychological distress of lung cancer patients during the perioperative period included physical problems, practical problems, medical expenses, emotional problems, and family communication problems. (1) The most significant factor in physical problems was respiratory status (*r* = 0.231, *P* < 0.001) while the most significant factor in emotional problems was anxiety (*r* = 0.415, *P* < 0.001). The reason for this may be that patients after lung cancer surgery have different degrees of respiratory restriction due to different surgical methods and individual physical differences. Because of this physical discomfort, the patient's internal psychological stress response may be manifested as persistent state of anxiety, fear, sadness, and other emotions, which in turn lead to different degrees of psychological pain experience. Therefore, medical staff should understand and pay attention to the psychological and physical health of patients, and provide them with multifaceted understanding and support. At the same time, it is also suggested that it is necessary to carry out health education on early pulmonary rehabilitation for lung cancer patients and to develop individualized intervention measures to improve patients' respiratory limitation, relieve physical discomfort, and improve psychological pleasure. (2) The most significant factor in actual problems is taking care of children (*r* = 0.228, *P* < 0.001), and the most significant factor in family communication problems is communication with parents (*r* = 0.151, *P* < 0.001). The most significant factor was work/study (*r* = 0.235, *P* < 0.001). The reason for the analysis of the above factors may be that lung cancer patients are in a period of role transition from healthy persons to patients at this time, and their social roles are changing, so they will face different role conflicts, leading to family life, work, and study. In addition, role conflict is closely related to mental health [19]. Anxiety and annoyance occur when a person is in a state of role conflict, and serious role conflict can also have a very negative impact on an individual's mental health. Studies have found that the psychosocial level of lung cancer patients is low, and their ability to cope with role conflicts is weak due to their incompetence or conflict with their original social role expectations [20], resulting in psychological and behavioral incompatibility and an inconsistent state. In the process of changing roles, many psychological problems are caused by an unclear understanding of roles. Medical staff can help lung cancer patients express their emotions and share their experiences through peer support and WeChat groups. Strategies to improve patients' cognition, help patients complete role transitions and reduce psychological pain caused by role conflicts. In addition to improving personal cognition, we should also pay attention to the role of family support. Studies have shown that [21] positive interaction and communication between medical staff and family caregivers can improve the quality of life of patients. Therefore, medical staff can work with family caregivers to formulate care plans for patients and provide real-time feedback, providing them with support for caring skills, emotional communication, disease management, etc., thereby improving the quality of life of patients.

The article "Analysis of Current Situation and Influencing Factors of Psychological Distress in Patients with Lung Cancer during Perioperative Period" was retracted in 2023. Reasons: unreliable results or conclusions; concerns about the data; concerns about the peer review; concerns about the citations.

### 5.4. Analysis of the Main Influencing Factors of Psychological Distress in Patients with Lung Cancer in the Perioperative Period

#### 5.4.1. Gender

The results of multiple regression analysis showed that the psychological distress score of female lung cancer patients was higher than that of male patients, which was consistent with previous research [22]. Data show that lung cancer deaths account for about 29.71% of all cancer death in men [1]. For women, lung cancer is still the most common cause of cancer death, and the top five causes of cancer deaths in women account for about 60.06% of all cancer deaths. Compared with males, female patients have higher mortality and poorer prognosis, which may be the main factors contributing to their higher psychological distress scores. Women's social problems are more prominent than men's, such as social role problems (mother, wife, daughter), family/caregiver conflicts, making women's psychological stress and psychological problems more serious and complex. More attention is paid to the mental health of women with lung cancer.

The article "Analysis of Current Situation and Influencing Factors of Psychological Distress in Patients with Lung Cancer during Perioperative Period" was retracted in 2023. Reasons: unreliable results or conclusions; concerns about the data; concerns about the peer review; concerns about the citations.

#### 5.4.2. Economic Burden due to Disease

The results of this study show that there are statistically significant differences in the psychological distress scores of the economic burden brought by different degrees of disease, and the psychological distress scores of patients with a heavy economic burden are higher. The high morbidity and mortality of lung cancer not only imposes a health burden on patients but also imposes a heavy economic burden on countless families due to a series of cost problems such as surgery, postoperative treatment, drug costs, hospitalization, and re-examination. Although medical insurance can reimburse part of it, the part that patients need to pay for themselves will still cause a lot of economic burden to the family. Due to the worry about the cost, the patient is under great psychological pressure and the degree of psychological pain is more severe.

#### 5.4.3. No Interest in Daily Activities

The results of this study also showed that lack of interest in daily activities was an independent influencing factor of psychological distress in lung cancer patients. According to psychologists, people's increased body activity will speed up blood circulation and increase the elasticity of blood vessels, which will help reduce the fatigue of the brain and improve self-efficacy, which will make people feel happy and happy [23]. Otherwise, it will cause psychological discomfort. Thus, medical staff can increase patient interest in the activity by interpreting positive cases of the beneficiaries of the activity or by developing personalized daily activities to help patients turn interest into practical action. Different guidance strategies should also be adopted for lung cancer patients with different disease stages, and studies have shown that there is no evidence or recommendation on physical activity in patients with advanced cancer [23].

## 6. Summaries

The detection rate of psychological distress in perioperative patients with lung cancer is high, and 55.6% of perioperative patients with lung cancer have moderate psychological distress, suggesting that medical staff should pay attention to the management of psychological distress in perioperative patients with lung cancer. While the number of morbidities, the economic burden caused by disease, and lack of interest in activities are the main influencing factors, it is also necessary to fully consider the patient's breathing problems, childcare, work/school, communication with parents, and other related factors, and take different angles as the starting point, reduces the level of psychological distress in patients with perioperative lung cancer. On the other hand, the survey subjects of this study are limited by geographical areas, and there are certain limitations, and there is no long-term follow-up on the dynamic level of subsequent psychological distress in patients with lung cancer in the perioperative period, and relevant longitudinal studies are carried out. The research team will follow-up on the above shortcomings. Further in-depth research is expected to provide corresponding guidance and a basis for the clinical care of patients with lung cancer.

The article "Analysis of Current Situation and Influencing Factors of Psychological Distress in Patients with Lung Cancer during Perioperative Period" was retracted in 2023. Reasons: unreliable results or conclusions; concerns about the data; concerns about the peer review; concerns about the citations.

## Figures and Tables

**Table 1:** Psychological pain scores of all patients.

Scores	Number of people (*n*)	Percentage
<4	165	44.35
≥4	207	55.65

**Table 2:** Univariate analysis of general data for psychological distress in 372 perioperative patients with lung cancer.

Indexes	Number of cases	Pain rating	*P* value
Gender	372	4.10 ± 2.88	0.001
Male	142	3.38 ± 3.03	
Female	230	4.39 ± 2.71	

Age			
＜40 year	43	4.30 ± 2.48	0.139
40–60 year	178	4.23 ± 2.93	
≥60 year	151	3.64 ± 2.89	

Smoking			
No	297	4.11 ± 2.75	0.127
Yes	75	3.55 ± 3.31	

Marital status			
Married	332	4.06 ± 2.93	0.375
Unmarried	8	4.63 ± 1.85	
Divorced	12	3.08 ± 2.31	
Widowed	20	3.25 ± 2.57	

With or without children			
No	20	4.15 ± 2.56	0.811
Yes	352	3.99 ± 2.90	

Family relationship			
Poor	4	6.25 ± 1.89	0.001
Common	80	4.94 ± 2.79	
Well	288	3.71 ± 2.85	

Educational level			
Graduate and above	18	4.50 ± 3.38	0.065
Undergraduate and college	133	4.53 ± 2.84	
High school and secondary school	106	3.74 ± 2.92	
Junior high school	66	3.65 ± 2.95	
Elementary school and below	49	3.43 ± 2.41	

Ethnic			
Han nationality	341	4.02 ± 2.88	0.696
Minority	31	3.81 ± 2.88	

Religious belief			
Have	360	4.01 ± 2.86	0.611
Not have	12	3.58 ± 3.37	

Place of residence			
City	236	4.18 ± 2.93	0.375
Couty	72	3.62 ± 2.64	
Township	18	3.33 ± 3.60	
Rural area	46	3.93 ± 2.64	

Living alone			
No	302	4.12 ± 2.89	0.088
Yes	70	3.47 ± 2.77	

Profession			
Worker	36	3.67 ± 2.76	0.384
Farmer	56	3.66 ± 2.82	
Administration staff	54	4.37 ± 2.91	
Medical staff	10	4.10 ± 2.03	
Merchants and self-employed	18	3.44 ± 2.98	
Technical staff	24	4.38 ± 3.72	
Unemployed or unemployed	15	5.33 ± 3.11	
Retired	109	3.72 ± 2.91	
Others	50	4.42 ± 2.42	

Payment of medical expenses			
At own expense	27	4.37 ± 2.83	0.835
At state expense	10	3.80 ± 3.08	
Medical insurance or commercial insurance	268	4.02 ± 2.84	
NCMS	67	3.79 ± 2.88	

Per capita monthly income			
＜¥ 1000	19	3.74 ± 2.71	0.582
¥ 1000–2999	77	4.13 ± 3.05	
¥ 3000–4999	137	3.83 ± 2.87	
¥ 5000–9999	86	3.87 ± 2.70	
≥¥ 10000	53	4.55 ± 3.00	

Economic burden of disease			
Light	29	2.62 ± 2.26	0.002
Common	232	3.88 ± 2.81	
Heavy	111	4.60 ± 2.88	

Primary caregiver			
Spouse	174	4.12 ± 3.03	0.106
Children	147	3.67 ± 2.72	
Parents	9	6.11 ± 2.21	
Relatives	37	4.30 ± 2.69	
Nanny	5	3.60 ± 3.05	

Character			
Outgoing	306	3.95 ± 2.41	0.056
Introverted	149	4.43 ± 2.61	

Current state			
Preoperative	195	3.38 ± 2.69	0.001
Postoperative	177	4.68 ± 2.92	

Incidence			
Initial onset	358	4.06 ± 2.89	0.047
Relapse	14	2.50 ± 2.18	

Number of lesions			
Single	219	4.19 ± 2.97	0.124
Multiple	153	3.73 ± 2.73	

Degree of obesity			
Lightweight	12	3.92 ± 1.67	0.869
Normal	175	4.08 ± 2.79	
Overweight	114	3.82 ± 2.94	
Obesity	71	4.11 ± 3.17	

Underlying disease			
Not have	266	3.95 ± 2.82	0.632
Have	106	4.11 ± 3.03	

Diabetes			
Not have	339	3.97 ± 2.86	0.527
Have	33	4.30 ± 3.10	

COPD			
Not have	370	4.00 ± 2.88	1
Have	2	4.00 ± 2.83	

Other diseases			
Not have	317	3.96 ± 2.83	0.478
Have	55	4.25 ± 3.15	

Whether the child is an adult			
No	75	4.21 ± 2.47	0.473
Yes	297	3.95 ± 2.97	

The article "Analysis of Current Situation and Influencing Factors of Psychological Distress in Patients with Lung Cancer during Perioperative Period" was retracted in 2023. Reasons: unreliable results or conclusions; concerns about the data; concerns about the peer review; concerns about the citations.

**Table 3:** Correlation analysis of psychological distress score and clinical factors in 372 perioperative patients with lung cancer.

Indexes	*r*	*P*
Physical problems		
Change in appearance	0.183	0.012
Surgical scar	0.169	<0.001
Bathing and dressing	0.092	0.075
Breathing condition	0.213	<0.001
Changes in urination	0.158	0.002
Indigestion	0.110	0.019
Memory/attention	0.180	<0.001
Mouth pain/ulcer	0.029	0.543
Nausea/Nausea	0.106	0.023
Nasal dryness/congestion	0.123	0.009
Constipate	0.168	0.001
Diarrhea	0.105	0.042
Eat	0.164	0.002
Tired	0.225	<0.001
Swelling of the limbs	0.118	0.023
Fever	0.144	0.006
Difficulty with activities after illness	0.257	<0.001
Pain	0.250	<0.001
Sexual desire/sexual function	0.056	0.282
Dry/itchy skin	0.036	0.486
Sleeping	0.289	<0.001
Tingling in hands and feet	0.117	0.024
Difficulty moving the arm	0.160	0.002

Practical problems		
Take care of children	0.228	<0.001
Housekeeping (housekeeping)	0.223	<0.001
Daily financial situation of the family	0.205	<0.001
degree of obesity	0.065	0.107
Quit smoking	0.110	0.408
Hypertension	0.032	0.268
Diabetes	0.026	0.309
COPD	0.008	0.436
Other diseases	0.040	0.223
Children of adulthood	0.085	0.052

Medical expenses		
Inconvenient to go out	0.187	<0.001
Work/study	0.235	<0.001
Lack of knowledge	0.126	0.015
Daily life is disrupted	0.223	<0.001

Emotional problems		
Depression	0.248	<0.001
Fear	0.317	<0.001
Sad	0.329	<0.001
Fear of recurrence	0.298	<0.001
Sad	0.343	<0.001
No interest in daily activities	0.281	<0.001
Complain	0.225	0.008
Easy to anger	0.291	<0.001
Psychological fragility	0.335	<0.001
Nervous	0.376	<0.001
Anxiety	0.415	<0.001
Guilty	0.202	<0.001
Lonely	0.219	0.020
Afraid	0.358	<0.001
Reliability	0.314	<0.001
Helplessness	0.260	<0.001
Social difficulties	0.214	<0.001
Family communication problems		
Communicate with husband and wife	0.147	0.005
Communicate with parents	0.151	0.003
Communicate with children	0.088	0.089
Have fertility problems	0.092	0.076

The article "Analysis of Current Situation and Influencing Factors of Psychological Distress in Patients with Lung Cancer during Perioperative Period" was retracted in 2023. Reasons: unreliable results or conclusions; concerns about the data; concerns about the peer review; concerns about the citations.

**Table 4:** Assignment table for logistic regression analysis.

Factors	Variables	Assignment
Gender	X1	Female = 0, male = 1
Economic burden of disease	X2	Light = 0, common = 1, heavy = 2
Take care of children	X3	Yes = 0, no = 1
Anxiety	X4	Continuous variable
No interest in daily activities	X5	Continuous variable

**Table 5:** Logistic regression analysis of psychological distress scores in 372 perioperative patients with lung cancer.

Variable	*β*	SE	Wald	*P*	OR	95% CI	
						Lower limit	Upper limit
Gender (male/female)	0.641	0.220	4.142	0.034	1.898	1.233	2.922
Economic burden of disease	0.702	0.214	6.347	0.01	2.018	1.327	3.069
Take care of children	1.343	0.685	3.977	0.042	3.831	1.001	14.667
Anxiety	1.086	0.444	4.207	0.026	2.962	1.241	7.073
No interest in daily activities	2.146	1.032	4.205	0.027	8.551	1.131	64.633

## Data Availability

The datasets used and/or analyzed during the current study are available from the corresponding author upon reasonable request.
